The article "Sustainable Energy Consumption Model for Textile Industry Using Fully Intuitionistic Fuzzy Optimization Approach" was published in 2022. Journal: Comput Intell Neurosci.

# Sustainable Energy Consumption Model for Textile Industry Using Fully Intuitionistic Fuzzy Optimization Approach

**DOI:** 10.1155/2022/5724825

**Published:** 2022-08-17

**Authors:** Sajida Kousar, Urooj Shafqat, Nasreen Kausar, Dragan Pamucar, Yeliz Karaca, Mohammed Abdullah Salman

**Affiliations:** ^1^Department of Mathematics and Statistics, International Islamic University Islamabad, Islamabad, Pakistan; ^2^Department of Mathematics, Faculty of Arts and Sciences Yildiz Technical University, Esenler 34210, Istanbul, Turkey; ^3^Faculty of Organizational Sciences, University of in Belgrade, Belgrade, Serbia; ^4^University of Massachusetts Medical School (UMASS), Worcester MA 01655, MA, USA; ^5^College of Education, Applied Sciences and Arts Amran University, Amran, Yemen

## Abstract

Consumption of renewable energy is on the rise because new technologies have made it cheaper and easier to meet the needs of a long-term energy source. In the present study, the idea of optimal usage of sustainable energy is discussed, taking into consideration the environmental and economic conditions that exist in Pakistan's textile manufacturing industry. By taking into account the regional potential for the application of renewable energy resources, solar energy generators are taken into consideration, and a fully intuitionistic fuzzy (FIF) textile energy model is constructed. Using the FIF model to determine the optimal distribution of solar energy units resulted in a tolerable number of unused energy units. These units may be returned to the central power supply station, which would save both money and energy.

## 1. Introduction

In the textile industry, electricity and thermal energy usage is the most common, as generated at industrial level through nonrenewable energy resources (petroleum, hydrocarbon gas liquids, natural gas, coal, etc.) or obtained directly through the government according to industrial policies. For example, in Pakistan, coal, nuclear, natural gas, hydroelectric, wind, and solar generators are the major electricity developing sources. Specifically, in Pakistan, the two crucial electricity producers are WAPDA (water and power development authority) that generates hydroelectricity and PEPCO (Pakistan electric power company) where distribution companies (DISCOs) under PEPCO work to maintain the path between electricity producers to consumer end by purchasing and selling it to representative area distribution companies. Except for one (K-electric), all these companies are owned by the government, and hence, the government provides different policies to different consuming sectors. In Pakistan, the energy crisis has been a never-ending situation from last two decades due to imbalance production and consumption ratio. At this point of energy crisis, the government of Pakistan and APTMA (All Pakistan Textile Mills Association) are on continuous conflict regarding the availability and favourable rates of energy. Working of textile industry is based on multiple stages like spinning, weaving, rewinding, dying, and so on, which are further subdivided into several other stages (see Figure 1).

All those stages require a huge amount of energy for their processing. Proper energy management planning can help industries to survive in natural crises or any other unpredictable conditions. Only if a single factor like energy optimization is focused, firstly, it will help industries to minimize their investing cost; secondly, the buyer will be able to get the product at a low cost. Thirdly, the saved energy will be used by other sectors like domestic sectors to fulfill their energy need and most importantly for the sake of healthy environmental and economic conditions, energy saving is a significant step. In the present time, when COVID-19 or other natural and economic disasters are happening, it is almost impossible to make an accurate and successful management plan. To ensure better energy management for textile industries under all these circumstances, developing an energy optimization model that can work in uncertain situations and generate the best optimal output is needed. To reduce the energy cost, one way is to reconsider the source of energy and replace it with the best convenient sustainable resource. Another way is to allocate energy units optimally. For the first way, considering the situation of Pakistan, it is best for textile industries to generate their own electricity and thermal energy through the Solar System. For the second way, it is best to modify the linear programming (LP) model for the textile industry according to the fuzzy environment. For this purpose, the conversion of the objective function, constraint equations, demand, and supply into fuzzy number is needed. Precisely that fuzzy number can overcome the uncertainty regarding material availability, working hours, financial and social barriers, labour, money, and space.

## 2. Literature Review

Although in Pakistan, textile industries cover 46% of the whole manufacturing sector and are a macro contributor with 8.5% of Pakistan's gross domestic product (GDP), it is also a huge environmental pollution contributor. In this setting, textile industries have a significant share in water and air pollution. The amount of clean water utilized by the textile industrial sector is substantially more as compared to the agricultural one [1], and for the production of one kg fabric output at the wet processing stage, the amount of water needed is almost 80–150 liters in addition to other chemicals [2]. Not only that, the report of 2015 stated that textile sector solely accounted for 1.2 billion tons of carbon dioxide [3], while according to the present behaviour of this industrial sector, 26% of carbon emission and 0.3 billion tons of crude oil consumption by the year 2025 is estimated by the study as well [3]. This is because the textile industry's fuel consumption is not only related to the production level but also during the transfer of textile products through different transportation means to different areas [4] taking part in carbon emission. All these aspects clear the reason for being called textile industry as the most polluting industry. In Faisalabad, Pakistan, a chain of textile industries is located around the road connecting twin districts Khuranwala and Jaranwala as shown in Figure 2.

Due to industrial water waste and carbon emission, the Khuranwala/Jaranwala road of 25–28 km long is full of unbearable smell and smog. The residents and daily travellers nearby face exposure to this unhealthy environment and suffer from breathing and eye diseases. By controlling abrupt energy consumption and ways connected to pollution either directly (industrial waste) or indirectly, like nonrecyclable fabric formation, excess of textile products, and so on, can help to lessen down pollution. Several studies have been conducted to reuse industrial water waste. Nadeem et al. [5] discussed the recycling and treatment potential of textile waste water by using membrane technology. According to Dehghani and Yoo [6], the organic components and approximate temperature of the textile industry's waste water are sufficient enough for the production of biofuel that can be used as a cheap source for creating thermal energy.

Efficient consumption of energy except proper planning is not possible in the region due to the complicated nature of the textile manufacturing sector. Spinning and weaving stages fully depend on electricity, while sizing, dying, and rewinding requires thermal energy to heat water or to dry the fabric [7, 8]. Studies have shown that, globally one trillion KWh of electricity is consumed per year to produce 60 billion kg fabric [9]. Usage of renewable energy resources like solar energy, geothermal energy, and landfill gas is helpful in the reduction of textile production costs. It lowers the total energy per unit usage that automatically degrade the environmental pollution factor as well. In Atlanta, seven textile manufacturing plants only use renewable electricity, and 89% of this electricity is renewable source [10].

Specifically, in Pakistan, the existence of energy self-sufficient textile industries is rare. The All Pakistan Textile Mills Association (APTMA) Punjab Chairman also insisted on adopting renewable solar energy resources to fulfill the need for electricity with affordable cost for the maintenance of industrial sustainability. According to their reporting, Pakistan textile industry is ready to shift to solar or hybrid energy generating systems [11]. This shift will not only reduce the cost but also reduce the carbon emission. In developing countries like Pakistan, where energy production is not proportional to the need, the cheap production and optimal allocation of energy is required. The usage of renewable energy resources can also be of great help for the industrial sector. Considering solar energy as a means for electricity is the best suitable option. The temperature and weather conditions of Pakistan as shown in Figure 3 can accelerate the outcome of the solar energy system.

The advancement of solar energy system makes electricity production much more efficient. Using this kind of system is considered as sustainable and ecological investment. Textile industry extensively uses electricity, so the optimal utilization of energy at each stage is regarded as an important initial target.

The conventional and most widely used method with reliable results for optimization is linear programming (LP) created by Kantorovich [13]. The only drawback of LP is its nonflexibility regarding nature. Natural scenarios are full of ambiguity, while classical optimization based on LP does not cover these uncertainties. After the revelation of fuzzy sets by Zadeh [14], LP also started to be modified. Zimmerman [15] used the concept of fuzziness in LP. He invented the technique to find a solution for fuzzy multiobjective LP. The fuzziness in this technique is due to the presence of fuzzy optimization conditions in it. Atanassov [16] improved the concept of fuzziness more by introducing a new generalization of a fuzzy set named intuitionistic fuzzy set, in which both the membership grade and nonmembership grade of element from decision set are necessary. This generalization created more optimization techniques [17]. Angelov [18] made the intuitionistic fuzzy LP technique. Subsequently, several researches has appeared on intuitionistic fuzzy linear programming (IFLP). Hussain and Kumar [19] worked on intuitionistic fuzzy transportation problem (IFTP). Ebrahimnejad and Verdegay [20] worked on a fully intuitionistic transportation problem (TP).

Several optimization models for sustainable production and consumption of renewable energy are constructed using bilevel programming [21], mixed integer linear programming [22], simulation-optimization modelling [23], linear programming [24–26], and goal programming [27] approach. Nematian and Farzi [28] considered the case study of energy recovered from urban solid waste in Iran and developed energy and environmental management model using fuzzy LP approach. Zhou et al. [29] used type-2 fuzzy chance-constrained fractional integrated modelling method for the management of energy system subjected to uncertainties and risks. Kouaissah and Hocine [30] and Hashemizadeh and Ju [31] introduced sustainable and renewable energy portfolios using a fuzzy interval goal programming technique. Khan et al. [32] examined and assessed the optimal cost system of electricity generation for the socio-economic sustainability of India by developing a sustainable and flexible electricity generation model using flexible fuzzy goal programming. Sustainable production in the textile industry depends upon the search of sustainable ways of energy management. Emeç and Akkaya [33] developed a fuzzy optimal renewable energy model (F-OREM) to solve the energy problem involving fuzzy parameters. Abbas et al. [34] systematically analyzed the potential of cotton crop waste to synergize industrial energy systems by integrating strategic and tactical decision models into an integrated model. The results indicate that cotton crop waste is a conducive and convenient source of sustainable energy supply for the textile industry. Techato et al. [35] presented a systematic review of the optimization models used in the textile industry, mostly established for cost minimization in logistics and production and optimized mainly with linear programming, integer programming, Markov chains, genetic algorithms, and multi-objective programming. The effectiveness of the present study in contrast with conventional LP is further discussed in upcoming sections where a fully intuitionistic fuzzy energy optimization model for Pakistan's textile industry is formed that results in optimal energy allocation that is further presented. For sustainability, the idea of replacing typical energy resources with solar energy generators along with its investing and working cost is also to be considered in reference to the existing self-sufficient textile industry of Pakistan.

## 3. Preliminaries

### 3.1. Intuitionistic Fuzzy Set

The intuitionistic fuzzy set was presented by Atanassov [16]; the degree of nonmembership and the degree of membership were expressed by the two characteristic functions. An intuitionistic fuzzy set (IFS) *𝒩* in 𝒬 can be described as an element of the following form *𝒩*={〈*s*, *ζ*_*𝒩*_(*s*), *η*_*𝒜*_(*s*)〉*|s* ∈ 𝒬} where the functions *η*_*𝒩*_ : 𝒬⟶[0,1] and *ζ*_*𝒩*_ : 𝒬⟶[0,1] represents the degree of nonmembership and the degree of membership of the component *s*  ∈  𝒬, respectively.

### 3.2. Triangular Intuitionistic Fuzzy Number

It is based on membership and nonmembership functions [36], considering $\tilde{Q_{l}^{⋎}}=\left(q_{1},q_{2},q_{3};{\overset{´}{q}}_{1},q_{2},{\overset{´}{q}}_{3}\right)$ such that ${\overset{´}{q}}_{1}\leq q_{1}\leq q_{2}\leq q_{3}\leq {\overset{´}{q}}_{3}$ and its membership function is defined as

(1) $$\begin{array}{c} \mu_{\tilde{Q_{l}^{⋎}}}=\left\{\begin{array}{cc} \frac{x-q_{2}}{q_{2}-q_{1}} & q_{1}\leq x<q_{2}\\ 1, & x=q_{2}\\ \frac{q_{3}-x}{q_{3}-q_{2}} & q_{2}<x\leq q_{3}\\ 0, & \text{otherwise}. \end{array}\right. \end{array}$$

The nonmembership function is as follows:

(2) $$\begin{array}{c} \nu_{\tilde{Q_{l}^{⋎}}}=\left\{\begin{array}{cc} \frac{q_{2}-x}{q_{2}-{\overset{´}{q}}_{1}} & {\overset{´}{q}}_{1}\leq x<q_{2}\\ 0, & x=q_{2}\\ \frac{x-q_{2}}{{\overset{´}{q}}_{3}-q_{2}} & q_{2}<x\leq {\overset{´}{q}}_{3}\\ 1, & \text{otherwise}. \end{array}\right. \end{array}$$

With restriction $0\leq \mu_{\tilde{Q_{l}^{⋎}}}x+\nu_{\tilde{Q_{l}^{⋎}}}x\leq 1$. If *q*_1_, *q*_2_, *q*_3_, ${\overset{´}{q}}_{1}$, and ${\overset{´}{q}}_{3}$ are nonnegative, then $\tilde{Q_{l}^{⋎}}$ will be a nonnegative intuitionistic fuzzy number. The geometrical interpretation of Triangular intuitionistic fuzzy number is presented in Figure 4.

### 3.3. Arithmetic Operations

Let $\tilde{Q_{l}^{⋎}}=\left(q_{1},q_{2},q_{3};{\overset{´}{q}}_{1},q_{2},{\overset{´}{q}}_{3}\right)$ and $\tilde{P_{l}^{⋎}}=\left(p_{1},p_{2},p_{3};{\overset{´}{p}}_{1},p_{2},{\overset{´}{p}}_{3}\right)$ are two triangular intuitionistic fuzzy numbers, then the algebraic operations between them are defined as follows:

1. $\tilde{Q_{l}^{⋎}}⊕\tilde{P_{l}^{⋎}}=\left(q_{1}+p_{1},q_{2}+p_{2},q_{3}+p_{3};{\overset{´}{q}}_{1}+{\overset{´}{p}}_{1},q_{2}+p_{2},{\overset{´}{q}}_{3}+{\overset{´}{p}}_{3}\right)$
2. $\tilde{Q_{l}^{⋎}}⊖\tilde{P_{l}^{⋎}}=\left(q_{1}-p_{3},q_{2}-p_{2},q_{3}-p_{1};{\overset{´}{q}}_{1}-{\overset{´}{p}}_{3},q_{2}-p_{2},{\overset{´}{q}}_{3}-{\overset{´}{p}}_{1}\right)$
3. $\kappa \tilde{Q_{l}^{⋎}}=\left(\kappa q_{1},\kappa q_{2},\kappa q_{3};\kappa {\overset{´}{q}}_{1},\kappa q_{2},\kappa {\overset{´}{q}}_{3}\right);for\kappa \geq 0$
4. $\kappa \tilde{Q_{l}^{⋎}}=\left(\kappa q_{3},\kappa q_{2},\alpha q_{1};\kappa {\overset{´}{q}}_{3},\kappa q_{2},\kappa {\overset{´}{q}}_{1}\right);for\kappa <0$
5. $\tilde{Q_{l}^{⋎}}⊛\tilde{P_{l}^{⋎}}=\left(r_{1},r_{2},r_{3};{\overset{´}{r}}_{1},r_{2},{\overset{´}{r}}_{3}\right)$

Here,

(3) $$\begin{array}{c} r_{1}=\min\left\{q_{1}p_{1},q_{1}p_{3},q_{3}p_{1},q_{3}p_{3}\right\}\\ r_{3}=\max\left\{q_{1}p_{1},q_{1}p_{3},q_{3}p_{1},q_{3}p_{3}\right\}\\ r_{2}=q_{2}p_{2}={\overset{´}{r}}_{2}\\ {\overset{´}{r}}_{1}=\min\left\{{\overset{´}{q}}_{1}{\overset{´}{p}}_{1},{\overset{´}{q}}_{1}{\overset{´}{p}}_{3},{\overset{´}{q}}_{3}{\overset{´}{p}}_{1},{\overset{´}{q}}_{3}{\overset{´}{p}}_{3}\right\}\\ {\overset{´}{r}}_{3}=\max\left\{{\overset{´}{q}}_{1}{\overset{´}{p}}_{1},{\overset{´}{q}}_{1}{\overset{´}{p}}_{3},{\overset{´}{q}}_{3}{\overset{´}{p}}_{1},{\overset{´}{q}}_{3}{\overset{´}{p}}_{3}\right\}. \end{array}$$

In particular, if $\tilde{Q_{l}^{⋎}}$ and $\tilde{P_{l}^{⋎}}$ are two nonnegative triangular intuitionistic fuzzy numbers, then their product $\tilde{Q_{l}^{⋎}}⊛\tilde{P_{l}^{⋎}}$ will be $\left\{q_{1}p_{1},q_{2}p_{2},q_{3}p_{3};{\overset{´}{q}}_{1}{\overset{´}{p}}_{1},q_{2}p_{2},{\overset{´}{q}}_{3}{\overset{´}{p}}_{3}\right\}$.

For the conversion of triangular intuitionistic fuzzy number into crisp following accuracy function [20] is used.

(4) $$\begin{array}{c} I\left(\tilde{Q_{l}^{⋎}}\right)=\frac{1}{8}\left(q_{1}+4q_{2}+q_{3}+{\overset{´}{q}}_{1}+{\overset{´}{q}}_{3}\right). \end{array}$$

## 4. Fully Intuitionistic Fuzzy Linear Programming Model

Mathematically, a general triangular fuzzy intuitionistic energy optimization model is expressed as follows:

(5) $$\begin{array}{c} \min\tilde{\alpha^{⋎}}=\sum_{j=1}^{m}\left\{\tilde{C_{j}^{⋎}}⊛\tilde{x_{j}^{⋎}}\right\}\\ \min\tilde{\alpha^{⋎}}=\left(\sum_{j=1}^{m}c_{j,1}x_{j,1},\sum_{j=1}^{m}c_{j,2}x_{j,2},\sum_{j=1}^{m}c_{j,3}x_{j,3};\sum_{j=1}^{m}{\overset{´}{c}}_{j,1}{\overset{´}{x}}_{j,1},\sum_{j=1}^{m}c_{j,2}x_{j,2},\sum_{j=1}^{m}{\overset{´}{c}}_{j,3}{\overset{´}{x}}_{j,3}\right). \end{array}$$

Subjected to triangular intuitionistic fuzzy energy optimization constraints,

(6) $$\begin{array}{c} \begin{array}{cc} \tilde{s_{21}^{⋎}}\tilde{x_{1}^{⋎}}+\tilde{s_{2j}^{⋎}}\tilde{x_{j}^{⋎}}+\cdots +\tilde{s_{2m}^{⋎}}\tilde{x_{m}^{⋎}}\; & \left(\leq =\geq \right)\;\tilde{D_{2}^{⋎}} \end{array}\\ \begin{array}{cc} \vdots \;\;\;\; & \left(\leq =\geq \right)\;\vdots \end{array}\\ \begin{array}{cc} \tilde{s_{n1}^{⋎}}\tilde{x_{1}^{⋎}}+\tilde{s_{nj}^{⋎}}\tilde{x_{j}^{⋎}}+\cdots +\tilde{s_{nm}^{⋎}}\tilde{x_{m}^{⋎}}\; & \left(\leq =\geq \right)\;\tilde{D_{n}^{⋎}} \end{array}\\ \tilde{s_{11}^{⋎}}\tilde{x_{1}^{⋎}}+\tilde{s_{1j}^{⋎}}\tilde{x_{j}^{⋎}}+\cdots +\tilde{s_{1m}^{⋎}}\tilde{x_{m}^{⋎}}\;\left(\leq =\geq \right)\;\tilde{D_{1}^{⋎}.} \end{array}$$

Here, $\tilde{x_{j}^{⋎}}\geq \tilde{0^{⋎}}$. The values of $\tilde{x_{j}^{⋎}}$ will optimize the intuitionistic fuzzy energy cost objective function where all the $\tilde{x_{j}^{⋎}}$ will satisfy the nonnegativity condition and constraint equations. In the above objective function $\tilde{C_{j}^{⋎}}=\left(c_{j,1},c_{j,2},c_{j,3};{\overset{´}{c}}_{j,1},c_{j,2},{\overset{´}{c}}_{j,3}\right)j=1,2,3,\ldots$ represent the triangular intuitionistic fuzzy cost coefficients and *s*_*ij*_ are the technological coefficients representing the amount of *i* th resource consuming at rate of $\tilde{x_{j}^{⋎}}$ per unit where

(7) $$\begin{array}{c} \tilde{D_{i}^{⋎}}=\left(d_{j,1},d_{j,2},d_{j,3};{\overset{´}{d}}_{j,1},d_{j,2},{\overset{´}{d}}_{j,3}\right) \end{array}$$

refers to the total availability of the *i* th triangular intuitionistic fuzzy resource. For the conversion of intuitionistic fuzzy energy optimization model into linear programming problem, the accuracy function is used as defined in (4). The following equation presents the defuzzified objective function.

(8) $$\begin{array}{c} \min\sum_{j=1}^{m}\left(c_{j,1}x_{j,1},c_{j,2}x_{j,2},c_{j,3}x_{j,3};{\overset{´}{c}}_{j,1}{\overset{´}{x}}_{j,1},c_{j,2}x_{j,2},{\overset{´}{c}}_{j,3}{\overset{´}{x}}_{j,3}\right)\\ =\min\left\{\frac{1}{8}\sum_{j=1}^{m}\left(c_{j,1}x_{j,1}+4c_{j,2}x_{j,2}+c_{j,3}x_{j,3}+{\overset{´}{c}}_{j,1}{\overset{´}{x}}_{j,1}+{\overset{´}{c}}_{j,3}{\overset{´}{x}}_{j,3}\right)\right... \end{array}$$

The above defined set of triangular intuitionistic constraints (6) can be rewritten as follows:

(9) $$\begin{array}{c} \sum_{j=1}^{m}s_{ij}x_{j,1}\left(\leq =\geq \right)d_{i,1}.\\ \sum_{j=1}^{m}s_{ij}x_{j,2}\left(\leq =\geq \right)d_{i,2}\\ \sum_{j=1}^{m}s_{ij}x_{j,3}\left(\leq =\geq \right)d_{i,3}\\ \sum_{j=1}^{m}s_{ij}{\overset{´}{x}}_{j,1}\left(\leq =\geq \right){\overset{´}{d}}_{i,1}\\ \sum_{j=1}^{m}s_{ij}{\overset{´}{x}}_{j,3}\left(\leq =\geq \right){\overset{´}{d}}_{i,3} \end{array}$$

The optimal solution of *x*_*j*,1_, *x*_*j*,2_, *x*_*j*,3_, ${\overset{´}{x}}_{j,1}$, and ${\overset{´}{x}}_{j,3}$ will be obtained by solving objective function (7) under constraints of (4).

## 5. Energy Optimization Model for Textile Industry

The textile industry is usually based on five stages which are further subdivided into several others. The main five stages are spinning, sizing, rewinding, weaving, and dyeing. Each stage's product (*x*_*i*_′*s*) forward lessens quantity to the next stage, that is, input < output always. For example, 97% of stage 2 product is further processed for next weaving stage, and remaining 3% goes to the rewinding stage whose product again becomes the input of stage 2. Considering minimum waste up to 7% for weaving stage, the material processed further is 93% of total *x*_3_, at the last stage, the wastage is approximately 4%. Considering a standard five stages textile model, the per month demand of stage *x*_1_, *x*_4_, and *x*_5_ products 400 units, 600 units, and 20,000 units. Per month total working hours are 720 hours [37]. The electricity cost per unit is 20.62 PKR/kWh, fuel oil is 85.68 PKR/litre, and LPG cost at the rate of 19.4103 PKR/litre [38, 39]. Energy cost for each stage is presented in Table 1.

The formulation of above model in intutitionistic fuzzy environment provided triangular intuitionistic fuzzy cost coefficients that represent the cost spent during production period as follows:

(10) $$\begin{array}{c} \tilde{C_{j}^{⋎}}=\left\{\tilde{C_{1}^{⋎}}=\left(46.55,51.55,56.55;41.55,51.55,61.55\right)\right.,\\ \tilde{C_{2}^{⋎}}=\left(19.5653,24.5653,29.5653;14.5653,24.5653,34.5653\right),\\ \tilde{\begin{array}{c} C_{3}^{⋎}=\left(36.24,41.24,46.24;31.24,41.24,51.24\right),\\ \tilde{\begin{array}{c} C_{4}^{⋎}=\left(10.465,15.465,20.465;5.465,15.465,25.465\right),\\ \tilde{\left.C_{5}^{⋎}=\left(172.892,177.892,182.892;167.892,177.892,187.892\right)\right\}} \end{array}} \end{array}}. \end{array}$$

The monthly triangular intuitionistic fuzzy production demand in kg for three products and total availability of working hours in a month are stated as follows:

(11) $$\begin{array}{c} \tilde{D_{i}^{⋎}}=\left\{\tilde{D_{1}^{⋎}=\left(350,400,450;300,400,500\right)}\right..\\ \tilde{D_{2}^{⋎}}=\left(550,600,650;500,600,700\right),\\ \tilde{\begin{array}{c} D_{3}^{⋎}=\left(19950,20000,20050;19900,20000,20100\right),\\ \tilde{\left.D_{4}^{⋎}=\left(670,720,770;620,720,820\right)\right\}} \end{array}} \end{array}$$

Mathematically, intuitionistic fuzzy energy optimization is framed as follows:

(12) $$\begin{array}{c} \min\tilde{\alpha^{⋎}}=\left(\sum_{j=1}^{m}\tilde{C_{j}^{⋎}}⊛\tilde{x_{j}^{⋎}}\right)=\left(\left(46.55,51.55,56.55;41.55,51.55,61.55\right)⊛\tilde{x_{1}^{⋎}}\right)\\ ⊕\left(\left(19.5653,24.5653,29.5653;14.5653,24.5653,34.5653\right)⊛\tilde{x_{2}^{⋎}}\right)\\ ⊕\left(\left(36.24,41.24,46.24;31.24,41.24,51.24\right)⊛\tilde{x_{3}^{⋎}}\right)\\ ⊕\left(\left(10.465,15.465,20.465;5.465,15.465,25.465\right)⊛\tilde{x_{4}^{⋎}}\right)\\ ⊕\left(\left(172.892,177.892,182.892;167.892,177.892,187.892\right)⊛\tilde{x_{5}^{⋎}}\right). \end{array}$$

Subject to

(13) $$\begin{array}{c} \tilde{x_{1}^{⋎}}⊖\tilde{x_{2}^{⋎}}\geq \left(350,400,450;300,400,500\right),\\ 0.03\tilde{x_{2}^{⋎}}⊖\tilde{x_{3}^{⋎}}⊕0.07\tilde{x_{4}^{⋎}}=\left(0,0,0;0,0,0\right),\\ 0.97\tilde{x_{2}^{⋎}}⊖\tilde{x_{4}^{⋎}}=\left(0,0,0;0,0,0\right),\\ 0.93\tilde{x_{4}^{⋎}}⊖\tilde{x_{5}^{⋎}}\geq \left(550,600,650;500,600,700\right),\\ 0.96\tilde{x_{5}^{⋎}}\geq \left(19950,20000,20050;19900,20000,20100\right),\\ 0.007\tilde{x_{1}^{⋎}}⊖0.007\tilde{x_{2}^{⋎}}⊕0.013\tilde{x_{4}^{⋎}}⊕0.0062\tilde{x_{5}^{⋎}}\leq \left(670,720,770;620,720,820\right),\\ \tilde{x_{i}^{⋎}}\geq \left(0,0,0;0,0,0\right),i=1,2,3,4,5, \end{array}$$

According to the above intuitionistic model, this formulated intuitionistic fuzzy energy optimization model is defuzzified as follows:

(14) $$\begin{array}{c} \min=\frac{1}{8}\left[46.55x_{1,1}+4\times 51.55x_{1,2}+56.55x_{1,3}+41.55{\overset{´}{x}}_{1,1}+61.55{\overset{´}{x}}_{1,3}\right]\\ +\frac{1}{8}\left[19.5653x_{2,1}+4\times 24.5653x_{2,2}+29.5653x_{2,3}+14.5653{\overset{´}{x}}_{2,1}+34.5653{\overset{´}{x}}_{2,3}\right]\\ +\frac{1}{8}\left[36.24x_{3,1}+4\times 41.24x_{3,2}+46.24x_{3,3}+31.24{\overset{´}{x}}_{3,1}+51.24{\overset{´}{x}}_{3,3}\right]\\ +\frac{1}{8}\left[10.465x_{4,1}+4\times 15.465x_{4,2}+20.465x_{4,3}+5.465{\overset{´}{x}}_{4,1}+25.465{\overset{´}{x}}_{4,3}\right]\\ +\frac{1}{8}\left[174.892x_{5,1}+4\times 177.892x_{5,2}+182.892x_{5,3}+167.892{\overset{´}{x}}_{5,1}+187.892{\overset{´}{x}}_{5,3}\right]. \end{array}$$

Subject to

(15) $$\begin{array}{c} x_{i,1}\geq 0,x_{i,2}\geq 0,x_{i,3}\geq 0,{\overset{´}{x}}_{i,1}\leq 0,{\overset{´}{x}}_{i,3}\leq 0wherei=1,2,3,4,5\\ 0.007x_{1,1}-0.007x_{2,3}+0.013x_{4,1}+0.0062x_{5,1}\leq 670,\\ 0.007x_{1,2}-0.007x_{2,2}+0.013x_{4,2}+0.0062x_{5,2}\leq 720,\\ 0.007x_{1,3}-0.007x_{2,1}+0.013x_{4,3}+0.0062x_{5,3}\leq 770,\\ 0.007{\overset{´}{x}}_{1,1}-0.007{\overset{´}{x}}_{2,3}+0.013{\overset{´}{x}}_{4,1}+0.0062{\overset{´}{x}}_{5,1}\leq 620,\\ 0.007{\overset{´}{x}}_{1,2}-0.007{\overset{´}{x}}_{2,2}+0.013{\overset{´}{x}}_{4,2}+0.0062{\overset{´}{x}}_{5,2}\leq 820,\\ x_{1,1}-x_{2,3}\geq 350,\\ x_{1,2}-x_{2,2}\geq 400,\\ x_{1,3}-x_{2,1}\geq 450,\\ 0.03x_{2,1}-x_{3,3}+0.07x_{4,1}=0,\\ 0.03x_{2,2}-x_{3,2}+0.07x_{4,2}=0,\\ 0.03x_{2,3}-x_{3,1}+0.07x_{4,3}=0,\\ 0.03{\overset{´}{x}}_{2,1}-{\overset{´}{x}}_{3,3}+0.07{\overset{´}{x}}_{4,1}=0,\\ 0.03{\overset{´}{x}}_{2,3}-{\overset{´}{x}}_{3,1}+0.07{\overset{´}{x}}_{4,3}=0,\\ {\overset{´}{x}}_{1,1}-{\overset{´}{x}}_{2,3}\geq 300,\\ {\overset{´}{x}}_{1,3}-{\overset{´}{x}}_{2,1}\geq 500,\\ 0.97x_{2,1}-x_{4,3}=0,\\ 0.97x_{2,2}-x_{4,2}=0,\\ 0.97x_{2,3}-x_{4,1}=0,\\ 0.97{\overset{´}{x}}_{2,1}-{\overset{´}{x}}_{4,3}=0,\\ 0.97{\overset{´}{x}}_{2,3}-{\overset{´}{x}}_{4,1}=0,\\ 0.93x_{4,1}-x_{5,3}\geq 550,\\ 0.93x_{4,2}-x_{5,2}\geq 600,\\ 0.93x_{4,3}-x_{5,1}\geq 650,\\ 0.93{\overset{´}{x}}_{4,1}-{\overset{´}{x}}_{5,3}\geq 500,\\ 0.93{\overset{´}{x}}_{4,3}-{\overset{´}{x}}_{5,1}\geq 700,\\ 0.96x_{5,1}\geq 19950,\\ 0.96x_{5,2}\geq 20000,\\ 0.96x_{5,3}\geq 20050,\\ 0.96{\overset{´}{x}}_{5,1}\geq 19900,\\ 0.96{\overset{´}{x}}_{5,3}\geq 20100. \end{array}$$

The optimal solution of (13) is

(16) $$\begin{array}{c} \tilde{x_{1}^{⋎}}=\left(24111.7,24159.4,24207.1;24064,24159.4,24254.8\right),\\ \tilde{x_{2}^{⋎}}=\left(23757.1,23759.4,23761.7;23754.8,23759.4,23764\right),\\ \tilde{x_{3}^{⋎}}=\left(874.161,874.107,874.054;874.125,874.107,874\right),\\ \tilde{x_{4}^{⋎}}=\left(23048.8,23046.6,23044.4;23051.1,23046.6,23024.1\right),\\ \tilde{x_{5}^{⋎}}=\left(20781.3,20833.3,20885.4;20729.2,20833.3,20937.5\right). \end{array}$$

By substituting the values of $\tilde{x_{i}^{⋎}}$'s in objective function (10), the minimal triangular intuitionistic fuzzy energy cost is calculated as follows:

(17) $$\begin{array}{c} \min\tilde{\alpha^{⋎}}=\left(\sum_{j=1}^{5}\tilde{C_{j}^{⋎}}⊛\tilde{x_{j}^{⋎}}\right)=\left(5463813.64,5927615.1,6403249.54;4979403.76,5927615.1,7880260.7\right)\\ \mu_{\tilde{Q_{l}^{⋎}}}\left(\tilde{\alpha^{⋎}}\right)=\left\{\begin{array}{cc} \frac{x-5927615.1}{5927615.1-5463813.64} & 5463813.64\leq x<5927615.1\\ 1, & x=5927615.1\\ \frac{6403249.54-x}{6403249.54-5463813.64} & 5927615.1<x\leq 6403249.54\\ 0, & \text{otherwise}, \end{array}\right.\\ \nu_{\tilde{Q_{l}^{⋎}}}\left(\tilde{\alpha^{⋎}}\right)=\left\{\begin{array}{cc} \frac{5927615.1-x}{5927615.1-4979403.76} & 4979403.76\leq x<5927615.1\\ 0, & x=5927615.1\\ \frac{x-5927615.1}{7880260.7-5927615.1} & 5927615.1<x\leq 7880260.7\\ 1, & \text{otherwise}. \end{array}\right. \end{array}$$

### 5.1. Postoptimal Analysis

Table 2 elaborates the flexibility of the presented model in intuitionistic fuzzy environment. Within the provided range for each variable, the model remains optimal and feasible. Since *x*_*i*_^*γ*^=(*x*_*i*,1_, *x*_*i*,2_, *x*_*i*,3_; *x*_*i*,1_′, *x*_*i*,2_, *x*_*i*,3_′); therefore, the allowable change in *x*_(*i*, *j*)_ will vast the range for *x*_*i*_^*γ*^ as well. This change will not impact the feasibility of the given model.

As shown in Table 3, the optimal results changed accordingly within the limits without impacting feasibility. The limit report of this model provided lower limit and upper limit for each decision variable along with its corresponding objective values. As the main objective is to minimize the energy cost, so here the optimal result is totally based on the lower limits to obtain minimum output. Whereas the upper limit is providing the range for feasible solution.  Table 4 presents the sensitivity report for the constraint equation. As there is not always perfect availability of resources and time so for each situation making new model is not possible. The following report allows us to predict the flexibility regarding the optimal and feasible results we could have obtained if the availability of resources fluctuate between the allowable increase and decrease.

### 5.2. Comparison

The solution of linear optimization problem under consideration is carried out by already existing linear programming (LP) and fuzzy linear programming techniques (FLP). The objective function value for the proposed method is less than LP and FLP techniques. The results are presented in Table 5.

From Figure 5, the degree of acceptance (rejection) of energy cost per month increases (decreases) from 5463813.64 to 5927615.1 and decrease (increases) from 5927615.1 to 6403249.54, while 5927615.1 is considered as required value where the level of acceptance is fully satisfied and degree of rejection is fully zero. The optimal solution of linear programming and fuzzy linear programming whose resulting cost are PKR 5987499 per month and 5980612.1 per month, while for proposed method it is 5927615.1 per month. This is evident that the fully intuitionistic fuzzy optimization model is more effectively minimize the energy cost as compared to linear programming approach.

## 6. Conclusion

Since Pakistan has a huge textile industrial sector and is now facing so many uncertainties due to the unpredicted policy shift 2020–25, therefore economically improving this sector will help every person belonging to the textile industry's hierarchy from consumers, labourers to stakeholder, and government. In Pakistan, government suggests industries to have a local supply of gas, which will create an explosion in production costs. According to the executive director of all Pakistan mills associations (APTAMA), the textile industry will face a 50% increase in the production cost [40]. The best option for Pakistan's industrial sector is to become self-sufficient as soon as possible. For this purpose, they need to change their habit of being dependent on the government for their energy resources. It is only possible to shift their energy modes from nonrenewable to renewable ones for sustainable energy production. According to regional temperature conditions of Pakistan as shown in Figure 2, solar energy production refines option. Since Pakistan's Kohinoor Textile Mills (KTML) in Rawalpindi, Pakistan, converted to a 6 Mw solar power plant with Reon energy making it affordable, sustainable, and more competitive. The implementation of this solar plant resulted in cost reduction and carbon footprint reduction. Because of its success, further three projects are also covered by KTML from 2017 to 2019, and their captive solar plant is saving almost 30% energy as well [41]. Therefore in Punjab, Pakistan, where there is a hub of textile industries should take a step forward towards the solar power plants.

The application of this solar plant project approximately requires 65 to 80 million in Pakistan. This project will contain a one Mw system that can produce 5000 units per day if minimum five hours of sunlight is considered. Monthly electricity unit production from this system will approximate between 150000 kWh and 180000 kWh. If LP solution is considered, the electricity unit per month consumed by all stages are 109108.6563 kWh and from FIFLP 106204.7783 kWh. In both cases, monthly electricity unit production through a solar plant is greater than need. The remaining electricity units can be sold out to the government or nearby industries that will accelerate to overcome the investing cost and the amount obtained from sold electricity can be further used for maintenance purpose as well. Decision making through FIFLP provide more flexible and optimal outputs. The less units industry will consume the more will be available for sale and soon the invested cost will overcome and providing profit. The conversion of few Pakistan's textile industry on solar power plants will help their neighboring industries, because the electricity cost per unit in solar generators is cheaper than other. That is, the government provide electricity at the rate of 20.62 Rs/Kwh while solar generating electricity cost is between 8 and 14 Rs/kWh.

The idea of intuitionistic fuzzy model helps in sufficient allocation of energy units that provides less wastage of energy. The implementation of this modelling can definitely lower down the production cost. For pilot study the implementation of sustainable energy optimization model on one of the industry from that region mentioned in Figure 1 can provide fruitful results along with the optimizing production cost of the neighboring industries as well.

## Figures and Tables

**Figure 1:** Textile industry processes.

**Figure 2:** Industrial chain of Khuranwala.

**Figure 3:** Temperature map of Pakistan (Pakistan Meteorological Department [12]).

**Figure 4:** Graphical representation of a triangular intuitionistic fuzzy number.

**Figure 5:** Graphical representation of LP, FLP, and FIF LP.

**Table 1:** Energy cost in PKR.

Energy	Spinning	Sizing	Weaving	Rewinding	Dyeing
Electricity	51.55	5.155	41.24	15.465	20.62
LPG	0	19.0103	0	0	135.8721
Furnace fuel	0	0	0	0	21.40
Total energy cost	51.55	24.5653	41.24	15.465	177.892

**Table 2:** Optimal feasible range.

Variable	Final value	Reduced cost	Objective	Allowable increase	Allowable decrease	Range
*x*_1,1_	24111.6857	0	5.819	1E + 30	5.819	5.819
*x*_1,2_	24159.37627	0	25.775	1E + 30	25.775	25.775
*x*_1,3_	24207.06684	0	7.069	1E + 30	7.069	7.069
*x*_1,1_′	24063.99512	0	5.194	1E + 30	5.194	5.194
*x*_1,3_′	24254.75742	0	7.694	1E + 30	7.694	7.694
*x*_2,1_	23757.06684	0	2.46	1E + 30	12.2144187	12.2144187
*x*_2,2_	23759.37627	0	12.283	1E + 30	46.3171348	46.3171348
*x*_2,3_	23761.6857	0	3.696	1E + 30	10.9589062	10.9589062
*x*_2,1_′	23754.75742	0	1.821	1E + 30	12.82117495	12.82117495
*x*_2,3_′	23763.99512	0	4.321	1E + 30	10.33814995	10.33814995
*x*_3,1_	874.1610548	0	4.53	1E + 30	365.2968733	365.2968733
*x*_3,2_	874.107453	0	20.62	1E + 30	1258.959902	1258.959902
*x*_3,3_	874.0538512	0	5.78	1E + 30	407.14729	407.14729
*x*_3,1_′	874.2146565	0	3.905	1E + 30	344.6049983	344.6049983
*x*_3,3_′	874.0002494	0	6.405	1E + 30	427.3724983	427.3724983
*x*_4,1_	23048.83513	0	1.308	1E + 30	11.29784144	11.29784144
*x*_4,2_	23046.59498	0	7.7325	1E + 30	47.74962351	47.74962351
*x*_4,3_	23044.35484	0	2.558	1E + 30	12.59218423	12.59218423
*x*_4,1_′	23051.07527	0	0.683	1E + 30	10.65788655	10.65788655
*x*_4,3_′	23042.1147	0	3.183	1E + 30	13.21770613	13.21770613
*x*_5,1_	20781.25	0	21.8615	1E + 30	35.40148304	35.40148304
*x*_5,2_	20833.33333	0	88.946	1E + 30	140.2896812	140.2896812
*x*_5,3_	20885.41667	0	22.8615	1E + 30	35.00971661	35.00971661
*x*_5,1_′	20729.16667	0	20.9865	1E + 30	35.19908724	35.19908724
*x*_5,3_′	20937.5	0	23.4865	1E + 30	34.94659306	34.94659306

**Table 3:** Limit report.

Variable	Final value	Lower limit	Objective value	Upper limit	Objective value
*x*_1,1_	24111.6857	24111.6857	5933823.792	58264.74189	6132560.426
*x*_1,2_	24159.37627	24159.37627	5933823.792	65363.31892	6995855.414
*x*_1,3_	24207.06684	24207.06684	5933823.792	72461.89595	6274937.179
*x*_1,1_′	24063.99512	24063.99512	5933823.792	51166.16486	6074592.462
*x*_1,3_′	24254.75742	24254.75742	5933823.792	79560.47298	6359345.968
*x*_2,1_	23757.06684	23757.06684	5933823.792	23757.06684	5933823.792
*x*_2,2_	23759.37627	23759.37627	5933823.792	23759.37627	5933823.792
*x*_2,3_	23761.6857	23761.6857	5933823.792	23761.6857	5933823.792
*x*_2,1_′	23754.75742	23754.75742	5933823.792	23754.75742	5933823.792
*x*_2,3_′	23763.99512	23763.99512	5933823.792	23763.99512	5933823.792
*x*_3,1_	874.1610548	874.1610548	5933823.792	874.1610548	5933823.792
*x*_3,2_	874.107453	874.107453	5933823.792	874.107453	5933823.792
*x*_3,3_	874.0538512	874.0538512	5933823.792	874.0538512	5933823.792
*x*_3,1_′	874.2146565	874.2146565	5933823.792	874.2146565	5933823.792
*x*_3,2_′	874.0002494	874.0002494	5933823.792	874.0002494	5933823.792
*x*_4,1_	23048.83513	23048.83513	5933823.792	23048.83513	5933823.792
*x*_4,2_	23046.59498	23046.59498	5933823.792	23046.59498	5933823.792
*x*_4,3_	23044.35484	23044.35484	5933823.792	23044.35484	5933823.792
*x*_4,1_′	23051.07527	23051.07527	5933823.792	23051.07527	5933823.792
*x*_4,3_′	23042.1147	23042.1147	5933823.792	23042.1147	5933823.792
*x*_5,1_	20781.25	20781.25	5933823.792	20781.25	5933823.792
*x*_5,2_	20833.33333	20833.33333	5933823.792	20833.33333	5933823.792
*x*_5,3_	20885.41667	20885.41667	5933823.792	20885.41667	5933823.792
*x*_5,1_′	20729.16667	20729.16667	5933823.792	20729.16667	5933823.792
*x*_5,3_′	20937.5	20937.5	5933823.792	20937.5	5933823.792

**Table 4:** Sensitivity report.

Constraint LHS	Final value	Shadow price	Constraint RHS	Allowable increase	Allowable decrease
1	430.9286066	0	670	1E + 30	239.0713934
2	431.5724014	0	720	1E + 30	288.4275986
3	432.2161962	0	770	1E + 30	337.7838038
4	430.2848118	0	620	1E + 30	189.7151882
5	432.859991	0	820	1E + 30	387.140009
6	350	5.819	350	34153.0562	24111.6857
7	400	25.775	400	41203.94265	24159.37627
8	450	7.069	450	48254.82911	24207.06684
9	300	5.194	300	27102.16974	24063.99512
10	500	7.694	500	55305.71557	24254.75742
11	−1.7053E-13	−5.78	0	874.0538512	1E + 30
12	−1.13687E-13	−20.62	0	874.107453	1E + 30
13	3.97904E-13	−4.53	0	874.1610548	1E + 30
14	−2.84217E-13	−6.405	0	874.0002494	1E + 30
15	2.27374E-13	−3.905	0	874.2146565	1E + 30
16	−7.27596E-12	10.00247423	0	1E + 30	23044.35484
17	−3.63798E-12	39.87278351	0	1E + 30	23046.59498
18	−7.27596E-12	9.949381443	0	1E + 30	23048.83513
19	−3.63798E-12	10.00737113	0	1E + 30	23042.1147
20	−3.63798E-12	9.930051546	0	1E + 30	23051.07527
21	19950	36.87654483	19950	23197.95231	19950
22	20000	146.1350846	20000	13722.05904	20000
23	20050	36.4684548	20050	16418.68769	20050
24	19900	36.66571588	19900	26587.58462	19900
25	20100	36.4027011	20100	13029.05538	20100
26	550	12.14821661	550	17102.79968	21435.41667
27	600	51.34368119	600	20633.66667	21433.33333
28	650	13.53998304	650	24164.53365	21431.25
29	500	11.46009306	500	13571.93269	21437.5
30	700	14.21258724	700	27695.40064	21429.16667
31	24111.6857	0	0	24111.6857	1E + 30
32	24159.37627	0	0	24159.37627	1E + 30
33	24207.06684	0	0	24207.06684	1E + 30
34	24063.99512	0	0	24063.99512	1E + 30
35	24254.75742	0	0	24254.75742	1E + 30
36	23757.06684	0	0	23757.06684	1E + 30
37	23759.37627	0	0	23759.37627	1E + 30
38	23761.6857	0	0	23761.6857	1E + 30
39	23754.75742	0	0	23754.75742	1E + 30
40	23763.99512	0	0	23763.99512	1E + 30
41	874.1610548	0	0	874.1610548	1E + 30
42	874.107453	0	0	874.107453	1E + 30
43	874.0538512	0	0	874.0538512	1E + 30
44	874.2146565	0	0	874.2146565	1E + 30
45	874.0002494	0	0	874.0002494	1E + 30
46	23048.83513	0	0	23048.83513	1E + 30
47	23046.59498	0	0	23046.59498	1E + 30
48	23044.35484	0	0	23044.35484	1E + 30
49	23051.07527	0	0	23051.07527	1E + 30
50	23042.1147	0	0	23042.1147	1E + 30
51	20781.25	0	0	20781.25	1E + 30
52	20833.33333	0	0	20833.33333	1E + 30
53	20885.41667	0	0	20885.41667	1E + 30
54	20729.16667	0	0	20729.16667	1E + 30
55	20937.5	0	0	20937.5	1E + 30

**Table 5:** Comparison of optimization techniques.

Variable	LP	FLP	FIF LP
*x*_1_	24195.38	(24126.743, 24159.376, 24192.008)	(24111.69, 24159.38, 24207.07; 24064, 24159.38, 24254.76)
*x*_2_	23759.38	(23736.743, 23759.376, 23782.008)	(23757.07, 23759.38, 223759.38; 23754.76,23759.38, 23764)
*x*_3_	2326.043	(2323.872, 2326.0429, 2328.2586)	(874.1611, 874.1075, 874.0539; 874.2147, 874.1075, 874.0002)
*x*_4_	23046.59	(23024.64, 23046.59, 23068.55)	(23048.84, 23046.59, 23044.35; 23051.08, 23046.59, 23042.11)
*x*_5_	20833.33	(20822.92, 20833.33, 20843.75)	(20781.25, 20833.33333, 20885.42; 20729.15, 20833.33333, 20937.5)
Objective function	5987499	5980612.1	5927615.1

## Data Availability

No data were used to support this study.
